# Antiulcer secondary metabolites from *Elaeocarpus grandis*, family Elaeocarpaceae, supported by *in silico* studies†

This article has been retracted.

**DOI:** 10.1039/d0ra06104b

**Published:** 2020-09-21

**Authors:** Radwa Taher Mohie El-Dien, Sherif A. Maher, Usama Ramadan Abdelmohsen, Asmaa M. AboulMagd, Mostafa Ahmed Fouad, Mohamed Salah Kamel

**Affiliations:** Department of Pharmacognosy, Faculty of Pharmacy, Deraya University University Zone 61111 New Minia City Egypt; Department of Biochemistry, Faculty of Pharmacy, Deraya University University Zone 61111 New Minia City Egypt; Department of Pharmacognosy, Faculty of Pharmacy, Minia University 61519 Minia Egypt usama.ramadan@mu.edu.eg; Department of Pharmaceutical Chemistry, Faculty of Pharmacy, Nahda University 62513 Beni Suef Egypt

## Abstract

*Elaeocarpus grandis* has a very potent analgesic effect, especially to a δ-opioid receptor, but its antiulcer activity has not yet been validated. Therefore, the present study was carried out to evaluate the antiulcer potential of the total methanolic extract and its derived fractions of the aerial parts of the plant using an indomethacin-induced gastric ulcer method. One new compound, grandisine H (1), and five known compounds, *P*-methoxy benzaldehyde, methyl gallate, kaempferol, quercetin and heterophyllin A (2–6), were isolated from the ethyl acetate fraction, which was the most potent one with an ulcer index value of 5 ± 1.95 (mm) ** (*P < 0.05, **P < 0.01) and a preventive index of 92.9%, following a bioassay-guided fractionation. The isolated compounds were subjected to a molecular docking study in an attempt to explain their significant antiulcer potential, and the results revealed that kaempferol and quercetin bind to the active site of the M3 receptor with a strong binding affinity *via* strong hydrogen bonds of −6.081 kcal mol^−1^ and −6.013 kcal mol^−1^, respectively. Also, quercetin and heterophyllin A showed a binding affinity with the gastric proton pump receptor and a strong hydrogen bond interaction with the amino acid active sites in the case of an H_2_-modeled receptor. These results clarify the effectiveness and importance of the ethyl acetate fraction as a natural anti-ulcer remedy.

## Abstract 2

*Elaeocarpus grandis* has a very potent analgesic effect, especially to a δ-opioid receptor, but its antiulcer activity has not yet been validated.

## 1. Introduction

Peptic ulcer are one of the most widely recognized gastrointestinal issues, which have a high prevalence in humans, especially in the inhabitants of developing nations.^1^ Peptic ulcer disorder, with its remissions and exacerbations, represents a public health problem.^2^ Additionally, it has been documented that approximately 10% of the population have or will develop a peptic ulcer.^3,4^ Ulcers occur due to an imbalance between aggressive factors (acid pepsin and *Helicobacter pylori*) and defensive factors (gastric mucus and bicarbonate secretion, prostaglandins, and innate resistance of the mucosal cells).^5^ A number of medications, including proton pump inhibitors, prostaglandin analogs, and histamine receptor antagonists are accessible for the treatment of peptic ulcers. However, a large portion of these medications produce several adverse effects, including toxicities and may even alter the biochemical mechanisms of the body with chronic usage.^6^ Hence, herbal medicines are commonly utilized in such situations when medications are to be used for long periods. Several natural drugs have been reported to possess antiulcerogenic activity by their overwhelming effect on mucosal defensive factors.^7,8^ (*e.g.*, those belonging to the Asteraceae, followed by the Combretaceae and Fabaceae families were reported to have promising antiulcerogenic activity *via* inhibition of gastric secretion and improvement in mucus secretion).^9^

*Elaeocarpus* is a genus of tropical and subtropical evergreen trees and shrubs belonging to the family Elaeocarpaceae. The family Elaeocarpaceae includes 40 species from five genera, *Aceratium*, *Dubouzetia*, *Elaeocarpaceae*, *Peripentadenia* and *Solanea*. The largest number of Elaeocarpaceae is in the genus *Elaeocarpus*, with 27 species.^10^ Furthermore, the family Elaeocarpaceae is found in the Australia-Pacific area, Asia including India and China, and Central and South America.^11^ Additionally, species from the genera *Elaeocarpus* and *Solanea* can be found from north Queensland to northern New South Wales. An estimated 400 species of Elaeocarpaceae from ten genera exist worldwide.^12^*Elaeocarpus* species contain various chemical constituents such as triterpenes,^13^ tannins,^14^ indolizidine alkaloids,^15,16^ rudrakine^17^ and flavonoids.^18^ Cordell *et al.*, in an elegant review of alkaloid-producing plant species, listed the family Elaeocarpaceae as a significant alkaloid-producing family, as grandisines A–G and (−)isoelaeocarpiline alkaloids were isolated from the leaves of *E. grandis*.^16,19,53^ Also, the number of other phytochemicals isolated from this family is very limited.^20^

Plants of the genus *Elaeocarpus* have been reported to be used in traditional medicines, particularly in India.^21^ Various *Elaeocarpus* species have also been widely studied for their pharmacological activities, such as analgesic,^22^ antifungal,^23^ antiinflammatory,^24,25^ antimicrobial,^26,27^ antidiabetic,^28^ antioxidant,^29,30^ antiviral,^31^ antitumor,^32^ antihypertensive,^33^ antianxiety^34^ and antidepressant activities.^35–37^

In our study, a bioassay-guided fractionation of the crude extract as well as histopathological investigation of antiulcer activity along with identification of phytoconstituents from the ethyl acetate fraction were performed.

## 2. Materials and methods

### 2.1 Chemicals and drugs

Silica gel G_60_F_254_ for thin-layer chromatography (TLC) was used for vacuum liquid chromatography (VLC, El-Nasr Company for Pharmaceuticals and Chemicals, Egypt), silica gel 60 for column chromatography (60–120 mesh, NICE and SDFCL SD Fine-Chem Limited, India), Sephadex LH-20 (GE Health Care, Sweden), precoated silica gel plates G_60_F_254_ plates (20 × 20 cm, 0.25 mm aluminum sheets, E-Merck, Germany), carboxymethylcellulose (El-Nasr Company for Pharmaceuticals and Chemicals (ADWIC), Egypt), normal saline 0.9% (El-Nasr Company for Pharmaceuticals and Chemicals (ADWIC), Egypt), indomethacin (Liometacin®, El-Nile Co., Egypt), ranitidine (Zantac®, GlaxoSmithKline (GSK), Egypt).

### 2.2 Experimental animals

Healthy adult male albino rats weighing about (200 ± 50 g each) were obtained from the animal house of the Faculties of Medicine of both Assuit and Minia Universities. The Institutional Animal Ethics Committee approved the protocol adopted for the experimentation on animals. All animal procedures were performed in accordance with the Guidelines for Care and Use of Laboratory Animals of Minia University and approved by the Animal Ethics Committee of the Institute (Approval reference number 57/2019). They were housed and bred under standardized environmental conditions (temperature 23 ± 2 °C and humidity 55 ± 15%) and fed with a standardized diet and water. Rats were deprived of food 24 hours before the experiment to ensure an empty stomach; but allowed free access to water; and kept in mesh-bottom cages to minimize coprophagia. Acclimatization for the experiment was done for one week before commencement of the experiment and all conditions were set to minimize animal suffering. All rats were employed in the experiment at the same time of the day to avoid variations due to diurnal rhythms as putative regulators of gastric functions.^38^

### 2.3 Plant material collection and identification

Aerial parts (leaves and stems) were taken from *Elaeocarpus grandis* L. cultivated in El-zohriya botanical garden, Cairo, Egypt. They were collected in December 2015 and kindly identified by Prof. Nasser Barakat, Professor of Botany, Department of Botany, Faculty of Science, Minia University, Minia, Egypt. A voucher specimen was deposited in the herbarium of the Pharmacognosy Department, Faculty of Pharmacy, Minia University, Minia, Egypt with the number [Mn-Ph-Cog-036].

### 2.4 Preparation of plant extract and fractionation

The air-dried powdered leaves and stems (2 kg) of *E. grandis* were extracted by maceration with 95% methanol until exhaustion. The alcoholic extract was concentrated under reduced pressure to a syrupy consistency (150 g), which was then suspended in the least amount of distilled water, transferred to a separating funnel and defatted with light petroleum ether. The total combined petroleum ether fractions were concentrated under reduced pressure to give fraction I (18.6 g). The mother liquor was then extracted with several portions of DCM. The combined DCM fractions were concentrated under reduced pressure to give fraction II (10.0 g). Finally, the remaining mother liquor was extracted with successive portions of ethyl acetate and the combined ethyl acetate fractions were concentrated under reduced pressure to give fraction III (40.0 g).

### 2.5 Determination of acute toxicity tests

An acute toxicity study of the total methanolic extract of *E. grandis* was performed by measuring the lethal dose for 50% of the laboratory animals (LD_50_ method),^39^ Different dose levels (0.5, 1, 1.5, 2, and 2.5 gm kg^−1^, p.o.) of the total methanolic extract (suspended in 0.5% CMC) were administered to different groups of rats (30 ± 5 g), containing six rats each. The control group received an equivalent dose of the total extract vehicle, 0.5% CMC solution. Both the test and control groups were observed for 48 h under normal environmental conditions, with free access to food and water.^40^

### 2.6 Grouping and dosing of animals

The experimental animals were randomly divided into seven groups, each containing six animals. Group (1) is the normal group receiving only the vehicle (0.5% CMC solution) with no administration of indomethacin. Group (2) is the −ve control group and it was given the vehicle (0.5% CMC solution). Group (3) is the +ve control group and it was given ranitidine 50 mg kg^−1^ p.o., and the other groups were administered the tested fractions at a dose level of 300 mg kg^−1^ p.o. (suspended in 0.5% CMC solution). After one hour, all groups except the normal group received a large dose of indomethacin (40 mg kg^−1^) orally to induce gastric ulceration.^41^ One hour later, all rats were sacrificed by cervical dislocation. The stomachs were removed, opened along their greater curvature, washed carefully with tap water and then with normal saline to remove gastric contents, and examined for macroscopic mucosal lesions.

### 2.7 Assessment of gastric mucosal lesions

Lesions were expressed in terms of the ulcer index (U.I.) which depends on calculation with the aid of an eye piece using a 0–3 scoring system based on the severity of each lesion. The severity factor was defined according to the length of the lesions. Severity factor 0 = no lesions; level 1 = lesions < 1 mm length; 2 = lesions 2–4 mm length and 3 = lesions > 4 mm length. The lesion score for each rat was calculated as the number of lesions in that rat multiplied by their respective severity factor. The U.I. for each group was taken as the mean lesion score of all rats in that group. The preventive index of a given drug was calculated using the following equation.^42^where P.I. is the preventive index and U.I. is the ulcer index.

### 2.8 Histological preparations for light electron microscopy (LEM)

A longitudinal section of the gastric tissue was taken from the glandular part of the stomach of each rat and fixed in a 10% formalin solution. After 24 h of fixation followed by embedding in a paraffin block, it was cut into sections of 5 micron onto a glass slide and stained with hematoxylin–eosin ready for examination.^42^

### 2.9 Statistical analysis

Data were expressed as mean ± standard error of mean (S.E.M) (*n* = 5). One-way analysis of variance (ANOVA) followed by Dunnett's test was applied. GraphPad Prism 5 was used for statistical calculations (GraphPad Software, San Diego, California, USA). The results were regarded as significant as follows: *P < 0.05, **P < 0.01, ***P < 0.001.

### 2.10 Molecular modeling studies

Molecular modeling studies were performed using MOE (Chemical Computing Group software, Canada). The 2D structures of the compounds were drawn using ChemDraw Ultra 11.0. The crystal structure of the M3 muscarinic acetylcholine receptor (PDB Entry Code 5ZHP)^43^ and gastrin proton pump (PDB Entry Code 5YLU)^44^ were extracted from the Brookhaven Protein Database (PDB: http://www.rcsb.org/pdb). As for the H-2 receptor, its 3D structure was created by homology modeling due to its unavailability in the protein data bank. During the docking process, all the enzyme crystal structures were checked for missing atoms and bonds. Energy minimization was established in the MMFF94x force field at a gradient value of 0.05. To guarantee the reliability of the docking process, redocking of the ligands into the binding site of the receptors was carried out. Consequently, the highest top conformation of ligands was generated by MOE and the results compared to the crystal structure-bound conformations. This procedure was performed three times in order to obtain reproducible results, and the RMSD between the docked ligand conformer and its target was less than 2. In this study, the docking protocol was selected as a docking program^45^ by applying proxy triangle methodology.^46^ The docked poses were ranked by an alpha HB scoring function, with refining and rescoring to remove the duplicate conformations in the same force field. At the end of the docking process, the lowest energy aligned conformation(s) were realized to analyze the binding affinity of the synthesized compounds and the three target receptors.

#### 2.10.1 Molecular descriptor analysis

Molecular descriptors of the isolated compounds were calculated using the “Calculate” module of MOE (Chemical Computing Group software, Canada). These parameters include MW, the number of hydrogen-bond acceptors (*a*_acc), the number of hydrogen-bond donors (*a*_don), an octanol/water partition coefficient (logP), the number of rotatable bonds (*B*_rotN), and the polar surface area (ASA_P).

#### 2.10.2 ADME studies

*In silico* ADME profiling was carried out using the online website “http://www.swissadme.ch/”. The calculated ADME parameters include BBB, GIT absorption, solubility, inhibition of CYP2D6, and bioavailability score.

## 3. Results and discussion

### 3.1 Phytochemical analysis

Because it displayed the highest antiulcer potential among the tested samples, the ethyl acetate fraction was fractionated into seven subfractions by VLC silica gel column chromatography using DCM–MeOH gradient mixtures in the order of increasing polarity. Subfraction 1 (6.0 g) was further fractionated using successive silica gel column chromatography using DCM–MeOH gradient mixtures to give compound 1 (10 mg) as an oily viscous liquid. Subfraction 2 (5.0 g) was further fractionated on a silica gel column to give four subfractions (f2a–f2d). Subfraction f2a was subjected to a Sephadex LH-20 column and purified by HPLC using H_2_O–MeOH (95 : 5) for 5 min, followed by a linear gradient to 100% MeOH within 30 min, and finally with a further isocratic elution with MeOH for 5 min at a flow rate of 2 ml min^−1^ to give compound 2 (100 mg; *R*_t_ = 14.387 min) while compound 3 (500 mg) was isolated by precipitation with methanol. Subfraction f2b (1.0 g) was subjected to a Sephadex LH-20 column using methanol 100% to give 3 subfractions (F2b_1_–F2b_3_). Subfractions F2b_1_ and F2b_2_ gave compounds 4 (500 mg) and 5 (280 mg), respectively, by precipitation. Subfraction 3 was added to subfraction 4 due to their similarity on TLC screening (yield 7.8 g) and subjected to a silica gel column, RP column chromatography and finally purified using a polyamide column to give compound 6.

#### 3.1.1 Identification of compounds

One new compound, grandisine H (1), and five known compounds were identified as,^15^*para*-methoxy benzaldehyde (2),^47^ methyl gallate (3),^48,49^ kaempferol (4),^50^ quercetin (5),^51^ and heterophyllin A (1,3-di-*O*-galloyl-4,6-hexahydroxydiphenoyl-α-d-glucopyranose) (6),^52^ as shown in Fig. 1.

**Fig. 1:** Compounds isolated from the ethyl acetate fraction of *E. grandis*.

Grandisine H compound 1 (10 mg) was isolated as an oily viscous liquid. Its molecular formula was determined to be C_16_H_22_NO_3_ as the HR-ESI-MS showed a significant quasi-M^+^ at = 276.1572 (found), 276.1521 (calcd) with an error of 0.0051 mm. The ^1^H NMR spectrum revealed that the upfield region consisted of a methyl doublet at *δ*_H_ 1.05 which was assigned to H-17, five multiplet methylene protons at *δ*_H_ 1.65, 1.82, 2.41, 2.14 and 2.75 which were assigned to H-1, H-2, H-13, H-14 and H-15, respectively, and one downfield shifted methylene proton at *δ*_H_ 3.49 which was assigned to H-3 due to attachment to a nitrogen group. Also, a doublet of doublet protons was observed at *δ*_H_ 2.93 with coupling constants *J* = 3.2 and 12 Hz which were assigned to H-8, one proton triplet at *δ*_H_ 3.37 (*J* = 7.5 Hz) assigned to proton H-6 and four multiplet methine protons at *δ*_H_ 4.65, 3.57, 3.54 and 1.16 which were assigned to H-5, H-7, H-9 and H-16, respectively. The downfield shifts of H-5 at *δ*_H_ 4.65 and H-6 at *δ*_H_ 3.37 were due to attached oxygen. The ^13^C-NMR spectrum showed 16 carbons, including one carbonyl carbon at *δ*_C_ 191.1 assigned to C-10, two quaternary carbons at *δ*_C_ 116.2 and 170.4 which were assigned to C-11 and C-12, and also the presence of a methyl carbon at *δ*_C_ 18.6 assigned to C-17, six methylenes at *δ*_C_ 34.1, 24.4, 58.6, 34.5, 24.7, 34.3 assigned to C-1, C-2, C-3, C-13, C-14, C-15, respectively, and six methines at *δ*_C_ 73.3, 55.0, 67.8, 45.7, 67.9, 20.4 assigned to C-5, C-6, C-7, C-8, C-9, C-16, respectively (Table 1).

**Table 1:** ^1^H, ^13^C and HMBC NMR spectral data of compound 1 (MeOD, 400 and 100 MHz)

Assignment	Chemical shift (*δ*_H_ ppm)	Multiplicity	*J* (Hz)	Chemical shift (*δ*_C_ ppm)	HMBC ^1^H to ^13^C
1	1.65	m	—	34.1	—
2	1.82	m	—	24.4	C-1, C-5
3	3.49	m	—	58.6	C-2, C-5
5	4.65	m	—	73.3	C-3, C-7
6	3.37	t	7.5	55.0	C-5, C-9
7	3.57	m	—	67.8	C-6
	Interchangeable with 9				
8	2.93	dd	3.2, 12	45.7	C-9, C-10
9	3.54	m	—	67.9	C-5
	Interchangeable with 7				
10	—	—	—	191.1	—
11	—	—	—	116.2	—
12	—	—	—	170.4	—
13	2.41	m	—	34.5	C-11, C-12, C-15
14	2.14	m	—	24.7	—
15	2.75	m	—	34.3	C-16, C-17, C-11, C-12
16	1.16	m	—	20.4	C-11, C-15, C-14
17	1.05	3H, d	6.84	18.6	C-11, C-15, C-16

Correlations observed in the heteronuclear multiple bond correlation spectroscopy (HMBC) spectrum allowed these partial structures to be connected. The indolizidine moiety was deduced from correlations between H-3 at *δ*_H_ 3.49 and C-9 and C-5 at *δ*_C_ 67.9 and 73.3, respectively. Also, between H-5 at *δ*_H_ 4.65 and C-9 at *δ*_C_ 67.9. The HMBC correlations between H-16 at *δ*_H_ 1.16 and the oxygenated quaternary carbon C-12 at *δ*_C_ 170.4 and the upfield quaternary carbon C-11 at *δ*_C_ 116.2 and between H-13 at *δ*_H_ 2.41 and C-12 and C-11 indicated that the two remaining partial structures were established (Fig. 2).^16^ The indolizidine proton H-8 at *δ*_H_ 2.93 showed correlation to the C-10 ketone carbonyl at *δ*_C_ 191.1, indicating that the dihydropyran was connected to the indolizidine by a ketone bridge between C-8 and C-10. The methyl group at proton H-17 *δ*_H_ 1.05 was confirmed to be attached to C-15, C-16 and an olefinic carbon C-11 at *δ*_C_ 34.3, 20.4 and 116.2 through HMBC correlations. The methylene proton H-15 at *δ*_H_ 2.75 also correlated to the methyl carbons C-17, C-11 and C-12 at *δ*_C_ 18.6, 116.2 and 170.4. With respect to the relative stereochemistry of compound 1, which was determined through the coupling constant of H-6 (t, *J* = 7.5 Hz), it indicated that H-6, H-5 and H-7 are axial. Additionally, the coupling constant of H-8 (dd, *J* = 3.2 and 12 Hz) indicated that H-8 should be axial, while H-9 is equatorial.

**Fig. 2:** Significant HMBC correlations of compound 1.

### 3.2 Antiulcer activity results

#### 3.2.1 Macroscopic results

Morphological investigation of the glandular part of the stomach of each rat revealed that indomethacin-treated stomachs showed marked gross mucosal damage, including tissue hyperaemia, different ulcer levels in the form of lines and spots, petechial lesions and hemorrhagic bands. Additionally, pretreatment with ranitidine, total extract and different fractions of *E. grandis* significantly reduced the gastric mucosal damage caused by indomethacin in the form of decreased hyperaemia, decreased ulcer formation and very mild or no petechial lesions, which are illustrated by Fig. 3, 4 and Table 2. It was observed that the lowest ulcer index with the maximum protection was achieved in rats pretreated with the ethyl acetate fraction, with a preventive index of 92.9%, followed by the DCM fraction with a preventive index of 90.1%, and all of them were more effective than ranitidine with a preventive index of 86.3%. They were followed by total extract and petroleum ether fractions with preventive indexes of 75.8% and 61.8%, respectively.

**Fig. 3:** Diagram representing the effect of indomethacin and its combination with other pretreatments on the ulcer index.

**Fig. 4:** Diagram representing the effect of indomethacin and its combination with other pretreatments on the preventive index of ulcers.

**Table 2:** Results of the effect of indomethacin on gastric lesions development and its alteration by various parameters^a^

Group	Level 1 lesions < 1 mm	Level II lesions 2–4 mm	Level III lesions > 4 mm	U.I. (mm)	P.I. (%)
Normal group	—	—	—	—	—
Indomethacin group (−ve control)	22.3 ± 0.7	15 ± 2.3	5.5 ± 1.2	70.2 ± 6.2	—
Indomethacin + ranitidine (+ve control)	4 ± 2.4	2 ± 0.4	0.2 ± 0.1	9.43 ± 0.3**	86.3
Indomethacin + total extract	4.68 ± 1	2.7 ± 0.07	2.9 ± 0.1	17 ± 0.22**	75.8
Indomethacin + petroleum ether fraction	5.8 ± 1.69	3 ± 1.14	5 ± 1.3	26.8 ± 5.9**	61.8
Indomethacin + DCM fraction	4.5 ± 0.21	1.5 ± 0.22	0.3 ± 0.44	7 ± 1.11**	90.1
Indomethacin + ethyl acetate fraction	3.1 ± 0.33	2.5 ± 4	0.4 ± 0.24	5 ± 1.95**	92.9

a All experimental groups were composed of 6 animals. The results of U.I. are expressed as the mean ± S.E. (standard error). Differences with respect to the control group were calculated using the Student's *T*-test (*P < 0.05, **P < 0.01). U.I. is the ulcer index and P.I. is the preventive index.

#### 3.2.2 Examination of the gross appearance of gastric mucosa from different groups

The gross appearance of gastric mucosa from the normal group appears normal with no mucosal injuries. Many ulcers of all levels, hyperaemia, haemorrhagic bands and dark brown petechial lesions were seen in the −ve control group. Those from the +ve control group show mild hyperaemia and ulcers mainly of level I. Furthermore, the group pretreated with total extract exhibited mild hyperaemia together with ulcers mainly of level I. The petroleum ether fraction group shows severe hyperaemia, petechial lesions and many ulcers mainly of level III. The DCM fraction group shows few ulcers mainly of level I. The gross appearance of gastric mucosa from the group pretreated with ethyl acetate fraction shows slightly congested tissue with very few ulcers of level I (Fig. 5).

**Fig. 5:** Gross appearance of gastric mucosa of different groups. Black arrows, ulcers; green arrows, hyperaemia; red arrows, haemorrhage.

#### 3.2.3 Histopathological results

Examinations of hematoxylin and eosin stained sections of the gastric mucosa from different rats of the normal group revealed a normal architecture formed of surface epithelium, lamina propria, and muscularis mucosa (Fig. 6a). The stomachs of rats from the +ve control group (treated with ranitidine) show submucosal oedema (small arrow), submucosal inflammatory cell infiltration (large arrow), and haemorrhage (arrow head) (Fig. 6b). Sections from group 1 (treated with total extract) show focal necrosis of gastric mucosa (small arrow), submucosal oedema (large arrow), and congestion of submucosal blood vessels (arrow head) (Fig. 6c). Those from group 2 (treated with the petroleum ether fraction) show congestion of mucosal blood vessels (small arrow) and submucosal inflammatory cell infiltration (large arrow) (Fig. 6d).

**Fig. 6:** (a–f) Histopathological appearance of gastric mucosa of different groups.

Sections from group 3 (treated with the DCM fraction) show focal necrosis of gastric mucosa (small arrow), congestion of submucosal blood vessels (large arrow) and submucosal oedema (arrow head) (Fig. 6e). The examined sections of group 4 (treated with the ethyl acetate fraction) showed less damage than the previous groups, expressed in normal intact mucosa, normal gastric pits, and lamina propria similar to those of the control group. However, there were slight submucosal oedema (small arrow) and submucosal infiltration with few inflammatory cells (large arrow) (Fig. 6f).

### 3.3 Docking study

For a better understanding of the significant antiulcer activity of the ethyl acetate fraction, the interactions between all the isolated compounds and the three receptors (M3, gastrin proton pump and H-2 receptor) were evaluated. The obtained docking poses revealed several hydrogen bonding and hydrophobic interactions with the key amino acids. The docked compounds were oriented approximately the same as the co-crystallized ligand, while the obtained interaction energies were comparable to that of the native ligand. The binding affinity energy of the poses and its orientation pose into the active site is chosen in a manner similar to the co-crystallized ligand orientation, taking into consideration the binding interactions, especially hydrogen bond and hydrophobic groups interactions.

The estimated binding score of the co-crystallized ligand of the M3 receptor (5ZHP) was −10.092 kcal mol^−1^ with complex hydrogen network interactions *via* a number of amino acids, including Ser 151 and Asn 507 and two hydrophobic interactions with Tyr 529 and Trp 503. Modeling studies suggest that compound 4 (kaempferol) binds to the active site of the M3 receptor with a binding affinity of −6.081 kcal mol^−1^*via* strong hydrogen bonding interaction of the phenolic hydroxyl groups with Tyr 529 and Thr 231 amino acids (Fig. 7 and Table 3). In addition, one hydrophobic interaction was observed with Tyr 506 residue. Compound 5 (quercetin) with a binding affinity of −6.013 kcal mol^−1^ binds with three hydrogen bond interactions with amino acid residues, Ala 238, Cys 532 and Tyr 529, in addition to hydrophobic interaction with Tyr 506. In the case of the gastrin proton pump (PDB code 5YLU), it is worth mentioning that quercetin with a binding affinity score of −6.418 kcal mol^−1^ forms one hydrogen bond donor with Glu 343 similar to the co-crystallized ligand and two additional hydrogen bond interactions with Ala 335 and Asn 792 amino acid residues. This is consistent with the predicted binding interaction of this compound with the M3 receptor. Also, the highest binding energy affinity of compound 6 (heterophyllin A) provided one hydrogen bond donor and another hydrogen bond acceptor with Glu 343 and Cys 813 residues, respectively, which may explain the significant antiulcer activity of *E. grandis*. Regarding H-2 receptor binding site residues, it was interesting to observe that quercetin binds to Glu 343 *via* hydrogen bond interaction with the OH group of the phenolic moiety. Furthermore, the results of docking of heterophyllin A, which forms two hydrogen bond interactions with Arg 143 and Glu 142 and one hydrophobic interaction with Ser 145 residue, confirm the antiulcer activity of this compound. Therefore, these results indicate that the significant activity of the mentioned isolated compounds possibly involved in antiulcer activity by inhibition of the mentioned receptors.

**Fig. 7:** Binding sites of compounds 4, 5 and 6 within crystal structure of M3 (PDB code 5ZHP), gastrin proton pump (PDB code 5YLU) and modeled H-2 receptor. (A and B) 2D and 3D models of kaempferol and quercetin into active site of M3 show some hydrogen bonding and hydrophobic interaction with important active site residues, respectively. (C and D) 2D and 3D models of compounds 5 and 6 into active site of gastrin proton pump show some hydrogen bonding and hydrophobic interaction with important active site residues, respectively. (E and F) Binding site of quercetin and heterophyllin A into modeled H-2 receptor, respectively.

**Table 3:** Ranking results of binding energy of the 6 natural isolated compounds with the three target receptors^a^

Compound name	Binding energy score		
	5ZHP	5YLU	Homologed H-2 receptor
1-Grandisine H	1.596	−5.867	−4.107
2-*P*-Methoxy benzaldehyde	−4.274	−4.519	−4.020
3-Methyl gallate	−5.106	−4.994	−3.867
4-Kaempferol	−6.081	−6.163	−4.892
5-Quercetin	−6.013	−6.418	−5.106
6-Heterophyllin A	13.930 (NA)	−6.042	−7.011

a The shown score is the mean of three consecutive runs.

#### 3.3.1 Homology modeling

The 3D structure of the H-2 receptor was obtained by a homology model, using Swiss model software (Fig. 8). The sequence identity of 92% with the 3D structure of the GPCR family (PDB code 6LN2) was used as a template for homology model generation. QMEAN scoring function and DFIRE were used to validate the model. Furthermore, graphical plots of ANOLEA mean force potential, GROMOS empirical force field energy and the neural network-based approach tools are considered in order to guarantee the correct modeling of the target protein. It was observed that both the target and the template indicated close structural identity, with RMSD values of 0.86 Å. This encouraged us to further use this model in this study.

**Fig. 8:** Generated homology model of H-2 receptor.

#### 3.3.2 Molecular descriptor analysis

An orally active compound should obey Lipinski's and Veber's rules, and the results shown in Table 4 for all the isolated compounds except heterophyllin A followed Lipinski's rule of five. Additionally, both grandisine H and *p*-methoxy benzaldehyde obey all Lipinski's and Veber's rules. Yet, compounds 3, 4, 5, and 6 which obey Veber's rule with one exception have a higher ASA_P value than the acceptable level. However, the overall drug-likeness properties are perfect, which emphasizes their potential to pass the drug development process.

**Table 4:** Compliance of the synthesized compounds to Lipinski's rule

Compound	logP(o/w) (<5)	MW (<500)	*a*_acc^a^ (≤10)	*a*_don^b^ (≤5)	*B*_rotN^c^ (≤10)	ASA_P^d^ (<140 Å)
1-Grandisine H	1.362	275.348	4	0	0	64.26
2-*p*-Methoxy benzaldehyde	1.789	136.150	2	0	2	101.192
3-Methyl gallate	0.993	184.147	4	3	2	197.301
4-Kaempferol	2.305	286.239	5	4	1	202.870
5-Quercetin	2.032	302.238	6	5	1	242.751
6-Heterophyllin A	2.566	786.560	18	13	6	612.515

a Number of hydrogen-bond acceptors (*a*_acc).

b Number of hydrogen-bond donors (*a*_don).

c Number of rotatable bonds (*B*_rotN).

d Polar surface area (ASA_P).

### 3.4 ADME studies

Moreover, all the isolated compounds were predicted and analyzed for pharmacokinetic properties, namely, blood–brain barrier (BBB) penetration, gastrointestinal absorption, solubility, inhibition of CYP2D6, and bioavailability.

The results showed that only compounds 1 and 2 showed good BBB penetration while the rest of the isolated compounds showed poor BBB penetration due to their high hydrophilicity. All compounds with the exception of heterophyllin A showed high GIT absorption and moderate water solubility. Regarding inhibition of CYP2D6, the results revealed that only kaempferol and quercetin could inhibit CYP2D6 while the bioavailability score range from 0.55 to 0.56 except for compound 6 (Table 5).

**Table 5:** Predicted ADME profiles of the synthesized compounds

Compound	BBB^a^	GIT absorption^b^	Solubility^c^	CYP2D6^d^	Bioavailability score^e^
1-Grandisine H	Yes	High	−2.32	No	0.56
2-*p*-Methoxy benzaldehyde	Yes	High	−3.97	No	0.56
3-Methyl gallate	No	High	−2.27	No	0.55
4-Kaempferol	No	High	−3.86	Yes	0.55
5-Quercetin	No	High	−3.91	Yes	0.55
6-Heterophyllin A	No	Low	−8.75	No	0.17

a Predicts the ability of the compound to penetrate the blood–brain barrier (BBB) according to the yolk of a boiled egg.

b Predicts gastrointestinal absorption according to the white of a boiled egg.

c Predicts the solubility of each compound in water. Levels <−10, <−6, <−4, <−2, <0 correspond to insoluble, poorly soluble, moderately soluble, soluble, very soluble, respectively.

d Predicts the cytochrome P450, 2D6 inhibition.

e Predicts the bioavailability score.

## 4. Conclusions

The present study revealed the antiulcer effect of the aerial parts of *E. grandis* methanolic extract and its derived fractions together with identification of six compounds from the ethyl acetate fraction as the most potent. The results showed that the ethyl acetate fraction possesses a potent *in vivo* antiulcer effect against indomethacin-induced gastric ulcers and has a higher preventive index (92.9%) in comparison with ranitidine (86.3%). Additional confirmation for the mechanism of action was obtained through *in silico* molecular modeling and ADME studies to compose an idea about how the components mainly contribute to the antiulcer activity.

Based on the results in this study, the *E. grandis* ethyl acetate fraction can be used as a safe herbal remedy for the treatment of ulcers with comparable potency to other medications, such as ranitidine, with a lower incidence rate of adverse effects.

## Conflicts of interest

The authors declare that they have no conflict of interest.

## Supplementary Material

RA-010-D0RA06104B-s001
